The article "Intelligent Disease Prediagnosis Only Based on Symptoms" was published in 2021. Journal: J Healthc Eng.

# Intelligent Disease Prediagnosis Only Based on Symptoms

**DOI:** 10.1155/2021/9963576

**Published:** 2021-07-31

**Authors:** Fangfang Luo, Xu Luo

**Affiliations:** ^1^School of Nursing, Zunyi Medical University, Zunyi 563000, China; ^2^Department of Information Engineering, Zunyi Medical University, Zunyi 563000, China

## Abstract

People often concern the relationships between symptoms and diseases when seeking medical advices. In this paper, medical data are divided into three copies, records related to main disease categories, records related to subclass disease types, and records of specific diseases firstly; then two disease recognition methods only based on symptoms for the main disease category identification, subclass disease type identification, and specific disease identification are given. In the methods, a neural network and a support vector machine (SVM) algorithms are adopted, respectively. In the method validation part, accuracy of the two diagnosis methods is tested and compared. Results show that automatic disease prediction only based on symptoms is possible for intelligent medical triage and common disease diagnosis.

## 1. Introduction

At present, there is shortage of per capita medical resources, and high-quality medical resources are concentrated in large cities and large hospitals. In China, many patients have strong health awareness, even if their symptoms are not serious; they also flock to large hospitals to seek quality medical services. Constraints and conflicts between medical resource supply and demand are a long-standing phenomenon.

In medical consultations, what people intuitively care about are the relationships between symptoms and diseases. Nowadays, many people provide symptoms online to obtain prediagnosis results, and their objective is to screen critical illnesses and seek an advice for further accurate medical treatment.

An intelligent information system, which can automatically perform prediagnosis based on the symptoms provided by patients, can alleviate the problem of medical resource shortage. In this paper, such diagnosis methods are proposed. Through these methods, preliminary diagnoses can be provided for specialized diseases, and it can help medical workers in areas having underdeveloped medical resources implement medical triage and provide consultation services for people who will seek precise treatment in big hospitals. Additionally, a common disease diagnosis service can be realized for people who can seek medical treatment by themselves.

## 2. Related Works

Computer aided diagnosis research has begun since the last century. Most intelligent disease diagnosis researches focus on a certain type disease or only a specific disease. The contents mostly are intelligent diagnosis using machine learning algorithms based on pathology data, influencing factors, examination data, physiological performance, or images when disease types are known previously [1–7]. Some exploratory works have discussed the disease diagnosis only based on the symptoms provided by patients. A simple method is to compare the symptoms provided by a patient to record symptoms in each data item, and the disease in the most similar entry is an output result. In [8], the user gives out feathers related to the diseases such as gender, age, affected part, and related symptoms firstly. Jackcard similarities are calculated based on symptom matrixes, and the similarities are arranged in descending order. Diseases in the first 3 items are selected as alternative recommended answers. In [9], the similarities, which are evaluated by differences between a symptom vector provided by the user and characteristic symptom sets of different diseases, are calculated. The similarities are also arranged in descending order, and the diseases in the first 3 selected items are alternative recommended answers. Disease diagnosis only based on symptoms and without disease type limitation is a general practice (GP) problem. If the above methods are used to solve this kind of diagnosis problem, the efficiency is extremely low, and repetition calculations are involved in each diagnosis case. In related works [10, 11], automatic disease diagnoses based on machine learning algorithms are proposed; in these works, symptoms are extracted firstly, and then, the diagnosis is implemented using deep learning algorithms. There are many diseases, while all proposed methods are limited to discussions on few diseases in the above papers.

The article "Intelligent Disease Prediagnosis Only Based on Symptoms" was published in 2021. Journal: J Healthc Eng.

Without detailed medical examination data and pathology support, accuracy of diagnosis methods based on symptoms cannot be guaranteed, while, in current online applications, reports, and documents, diagnosis only based on symptoms can be a disease screening method and used to help fast disease type recognition and disease triage in hospital. The key problem is the adaptability of this kind of diagnosis methods. At present, there is no discussion about which disease type levels or which diseases this kind of diagnosis methods is suitable for. To fill this gap, in this paper, this issue is considered.

Disease prediagnosis based on symptoms, which are contained in consultation words, is indeed a text classification problem. In these works, the first step would mostly be lexical feather extraction, and then classification based on different feather properties is implemented [12–14]. Considering the particularity in clinic and immature Chinese word segmentations, in this paper, we only discuss the core prediagnosis problem, and the symptoms, which are also disease feathers, have been extracted according to clinical experience previously. A hierarchical frame is provided in this paper. Firstly, the diseases are divided into major categories and then are divided into several subtypes. Furthermore, specific diseases are filled into subclass disease types. In this paper, two automatic diagnosis methods using a neural network technology and a support vector machine (SVM) technology, respectively, are given to solve this general practice (GP) problem. In the methods, the first is the major disease category identification, and then it is based on the results to identify disease subtypes. Further process is the training for specific disease identification. To observe the effectiveness, the two diagnosis methods are tested and compared.

## 3. Problem Statement and Theories in This Paper

### 3.1. The Diagnosis Problem in This Paper

The intelligent diagnosis problem to be solved in this paper includes two aspects. The first one is seeking diagnosis experience according to the relationships between symptoms and diseases. Here, supervised machine learning methods are adopted. The second one is disease prediction based on the symptoms provided by visitors. The first one is the main problem.

In our research, symptoms have been extracted in data preprocessing. Consider that samples with respect to the same disease type are in a hyperplane and linearly separable, and a different symptom may make two similar samples refer to different disease types; the support vector machine (SVM) algorithm is an appropriate method. As the neural network is a generic method in multiclassification problems, this method is also adopted in this paper and compared with SVM [15].

### 3.2. The Neural Network in This Paper

To describe this method, symbolic notations are given firstly:

 
*N*: there are *N* symptoms in each data item
 
Γ: the number of nodes in the output layer of a neural network
 
*Y*: the number of nodes in the hidden layer of a neural network is *Y*, and $Y=10+\sqrt{N+T}$
 
*hn*=(*hn*_1_, *hn*_2_, *hn*_3_,…, *hn*_*Y*_): the input vector of the hidden layer is *hn*, and the input of the *p*th hidden layer unit is *hn*_*p*_
 
*ho*=(*ho*_1_, *ho*_2_, *ho*_3_,…, *ho*_*Y*_): the output vector of the hidden layer is *ho*, and the output of the *p*th hidden layer unit is *ho*_*P*_
 
*yn*=(*yn*_1_, *yn*_2_, *yn*_3_,…, *yn*_Γ_): the input vector of the output layer is *yn*, and the input of the *q*th output layer unit is *yn*_*q*_
 
*yo*=(*yo*_1_, *yo*_2_, *yo*_3_,…, *yo*_Γ_): the output vector of the output layer is *yo*, and the output of the *q*th output layer unit is *yo*_*q*_
 
*w*_*np*_: the connection weight between the *n*th input layer unit and the *p*th hidden layer unit
 
*ϖ*_*pq*_: the connection weight between the *p*th hidden layer unit and the *q*th output layer unit
 
*b*_*p*_: the threshold value of the *p*th hidden layer
 
*b*_*q*_: the threshold value of the *q*th output layer
 
*x*_*k*_=(*x*_1_^(*k*)^, *x*_2_^(*k*)^,…, *x*_*N*_^(*k*)^): the *k*th symptom record, which contains *N* components, is *x*_*k*_, and each component represents a different symptom
 
*d*_*k*_=(*d*_1_^(*k*)^, *d*_2_^(*k*)^,…, *d*_Γ_^(*k*)^): the expected output when *x*_*k*_ is input to the neural network is *d*_*k*_, and if this record is about the *r* th disease or disease type, the component *d*_*r*_^(*k*)^=1, other components *d*_*j*_^(*k*)^=0(*j* ≠ *r*, *j* ∈ {1,2,3,…, Γ})
 
*o*(*k*)=(*x*_*k*_, *d*_*k*_)=((*x*_1_^(*k*)^, *x*_2_^(*k*)^,…, *x*_*N*_^(*k*)^), (*d*_1_^(*k*)^, *d*_2_^(*k*)^,…, *d*_Γ_^(*k*)^)): represents the *k*th training sample

In the neural network, each nerve cell is actually an activation function. For the *p*th hidden layer unit, if sample *o*(*k*) is used, the input is

(1) $$\begin{array}{c} hn_{p}^{\left(k\right)}=\sum_{n=1}^{N}w_{np}x_{n}^{\left(k\right)}-b_{p}. \end{array}$$

A sigmoid function is used as the activation function, and the output is

(2) $$\begin{array}{c} h{\left(k\right)}_{p}^{\left(k\right)}=f\left(hn_{p}^{\left(k\right)}\right)=\frac{1}{\left(1+\exp\left(-hn_{p}^{\left(k\right)}\right)\right)}, \end{array}$$

where exp() is an exponential function. An output cell of the hidden layer is an input cell of the output layer, and for the *q*th output layer unit, if sample *o*(*k*) is used, the input is

(3) $$\begin{array}{c} yn_{q}^{\left(k\right)}=\sum_{p=1}^{Y}\varpi_{pq}ho_{p}^{\left(k\right)}-\theta_{q}, \end{array}$$

and a softmax output is

(4) $$\begin{array}{c} y{\left(k\right)}_{q}^{\left(k\right)}=f_{2}\left(yn_{q}^{\left(k\right)}\right)=\frac{\exp\left(yn_{q}^{\left(k\right)}\right)}{\sum_{q=1}^{\Gamma }\exp\left(yn_{q}^{\left(k\right)}\right)}. \end{array}$$

Furthermore, in the neural network, a cross-entropy loss function is adopted:

(5) $$\begin{array}{c} e^{\left(k\right)}=f_{3}\left(yo_{q}^{\left(k\right)}\right)=-\sum_{q=1}^{\Gamma }d_{q}^{\left(k\right)}\ln y{\left(k\right)}_{q}^{\left(k\right)}. \end{array}$$

In the neural network, some important differential equations are also involved. The first is the partial differential of error function *e*^(*k*)^ with respect to *ϖ*_*pq*_, and it is

(6) $$\begin{array}{c} \frac{\partial e^{\left(k\right)}}{\partial \varpi_{pq}}=\frac{\partial e^{\left(k\right)}}{\partial yn_{q}^{\left(k\right)}}\cdot \frac{\partial yn_{q}^{\left(k\right)}}{\partial \varpi_{pq}}. \end{array}$$

Considering formula (3) and that the processing procedure is focused on the connection weight between the *p*th specific hidden layer unit and the *q*th specific output layer unit, the following formula can be obtained:

(7) $$\begin{array}{c} \frac{\partial yn_{q}^{\left(k\right)}}{\partial \varpi_{pq}}=\frac{\partial \left(\sum_{p=1}^{Y}\varpi_{pq}h{\left(k\right)}_{p}^{\left(k\right)}-\theta_{q}\right)}{\partial \varpi_{pq}}=ho_{p}^{\left(k\right)}. \end{array}$$

Further, based on formulas (4) and (5), there is

(8) $$\begin{array}{c} \frac{\partial e^{\left(k\right)}}{\partial yn_{q}^{\left(k\right)}}=\frac{\partial e^{\left(k\right)}}{\partial y{ο}_{q}^{\left(k\right)}}\cdot \frac{\partial y{ο}_{q}^{\left(k\right)}}{\partial yn_{q}^{\left(k\right)}}=-d_{q}^{\left(k\right)}+y{\left(k\right)}_{q}^{\left(k\right)}\sum_{q=1}^{\Gamma }d_{q}^{\left(k\right)}. \end{array}$$

Here, this result is marked as  *δ*_*q*_^(*k*)^.

The article "Intelligent Disease Prediagnosis Only Based on Symptoms" was published in 2021. Journal: J Healthc Eng.

If *δ*_*q*_^(*k*)^ is obtained, it can be used to renew the weight between a hidden layer unit and an output layer unit, and the update rule is

(9) $$\begin{array}{c} \varpi_{pq}=\varpi_{pq}+\eta \frac{\partial e^{\left(k\right)}}{\partial \varpi_{pq}}=\varpi_{pq}+\eta \delta_{q}^{\left(k\right)}h{\left(k\right)}_{p}^{\left(k\right)}. \end{array}$$

The connection weight between the *p*th hidden layer unit and the *q*th output layer unit in the next training process is the connection weight at present combined with the partial differential *δ*_*q*_^(*k*)^ and output *ho*_*p*_^(*k*)^. *η* is a given learning rate.

In the concrete implementation process, the parameter values of *k*, *p*, and *q* are given in operations with respect to a particular neuron unit.

In the neural network, the partial differential of error function *e*^(*k*)^ with respect to *w*_*np*_ is also involved, and it is shown as follows:

(10) $$\begin{array}{c} \;\frac{\partial e^{\left(k\right)}}{\partial w_{np}}=\frac{\partial e^{\left(k\right)}}{\partial h{\left(k\right)}_{p}^{\left(k\right)}}\cdot \frac{\partial hn_{p}^{\left(k\right)}}{\partial w_{np}}. \end{array}$$

Similarly, considering formula (2) and that the processing procedure is focused on the connection weight between the *n*th specific input layer unit and the *p*th specific hidden layer unit, the following formula can be obtained:

(11) $$\begin{array}{c} \frac{\partial hn_{p}^{\left(k\right)}}{\partial w_{np}}=\frac{\partial \left(\sum_{i=1}^{N}w_{np}x_{n}^{\left(k\right)}-b_{p}\right)}{\partial w_{np}}=x_{n}^{\left(k\right)}. \end{array}$$

Further, based on formulas (2)–(5), there is

(12) $$\begin{array}{c} \frac{\partial e^{\left(k\right)}}{\partial hn_{p}^{\left(k\right)}}=\frac{\partial e^{\left(k\right)}}{\partial yn_{q}^{\left(k\right)}}\cdot \frac{\partial yn_{q}^{\left(k\right)}}{\partial ho_{p}^{\left(k\right)}}\cdot \frac{\partial ho_{p}^{\left(k\right)}}{\partial hn_{p}^{\left(k\right)}}=-\left(\sum_{q=1}^{\Gamma }\delta_{q}^{\left(k\right)}\varpi_{pq}\right)f_{1}^{\prime }\left(hn_{p}^{\left(k\right)}\right),\\ =-\left(\sum_{q=1}^{\Gamma }\delta_{q}^{\left(k\right)}\varpi_{pq}\right)\exp\left(-hn_{p}^{\left(k\right)}\right){\left(1+\exp\left(-hn_{p}^{\left(k\right)}\right)\right)}^{-2}. \end{array}$$

Here, this result is marked as *σ*_*p*_^(*k*)^.

The article "Intelligent Disease Prediagnosis Only Based on Symptoms" was published in 2021. Journal: J Healthc Eng.

If *σ*_*p*_^(*k*)^ is obtained, it can be used to renew the weight between a hidden layer unit and an output layer unit, and the update rule is

(13) $$\begin{array}{c} w_{np}=w_{np}+\eta \frac{\partial e^{\left(k\right)}}{\partial w_{np}}=w_{np}+\eta \sigma_{p}^{\left(k\right)}x_{n}^{\left(k\right)}. \end{array}$$

The connection weight between the *n*th hidden layer unit and the *p*th output layer unit in the next training process is the connection weight at present combined with the partial differential *σ*_*p*_^(*k*)^ and input  *x*_*n*_^(*k*)^. *η* is also a given learning rate.

### 3.3. The Support Vector Machine (SVM) in This Paper

In this paper, a disease sample is *x*^(*k*)^=(*x*_1_^(*k*)^, *x*_2_^(*k*)^,…, *x*_*N*_^(*k*)^, *x*_*N*+1_^(*k*)^), where (*x*_1_^(*k*)^, *x*_2_^(*k*)^,…, *x*_*N*_^(*k*)^) represents different symptoms and *x*_*N*+1_^(*k*)^ is a disease or disease type.

The hyperplane separating samples are depicted as follows:

(14) $$\begin{array}{c} f\left(x\right)=\omega^{T}x+c. \end{array}$$

The purpose is to get the classification parameters **ω** and *c*. If there are *T*(*b*) samples in the sample space, the specific problem should be solved:

(15) $$\begin{array}{c} \underset{\left(\omega ,c\right)}{\min}\frac{1}{2}{\left\|\omega \right\|}^{2},\\ \text{s.t. }x_{N+1}^{\left(k\right)}\left(\omega {\left[x_{1}^{\left(k\right)},\ldots ,x_{N}^{\left(k\right)}\right]}^{T}+c\right)\geq 1,\;k=1,2,\ldots ,T\left(b\right). \end{array}$$

If the classification parameters have been obtained, and there is a symptom vector **k**=(*κ*_1_, *κ*_2_,…, *κ*_*N*_), while

(16) $$\begin{array}{c} \omega \kappa +c=\omega_{1}\kappa_{1}+\omega_{2}\kappa_{2}+\cdots +\omega_{N}\kappa_{N}+c>0, \end{array}$$

it can be determined that *κ* belongs to the disease category I, while

(17) $$\begin{array}{c} \omega \kappa +c=\omega_{1}\kappa_{1}+\omega_{2}\kappa_{2}+\cdots +\omega_{N}\kappa_{N}+c<0, \end{array}$$

and it can be determined that **κ** does not belong to the disease category I.

The article "Intelligent Disease Prediagnosis Only Based on Symptoms" was published in 2021. Journal: J Healthc Eng.

In learning procedures, a one-against-the-rest SVM method [16] based on this basic form can be adopted to implement multiclassification.

## 4. Disease Identification Methods

### 4.1. Preconditions

Suppose that a preprocess step has been implemented on existing electronic medical records. Disease symptoms, disease types, and relations between the two are known clearly.

### 4.2. Labelling

Number the *N* disease symptoms in the database, and the symptoms are numbered as 1,2,3,4,…, *N*, respectively. Considering that the same symptoms in different gender patients are often with regard to different common diseases or disease types, gender is deemed as a default “symptom,” which is labelled 1. Diseases in the database are divided into *B* main categories, which are numbered as *N∗*10+1, *N∗*10+2,…, *N∗*10+*B*. Each main disease category is further divided into several subclasses and numbered. There are *T*(*b*) subtype diseases under the main disease category *N∗*10+*b*, and they are numbered as *N∗*10+*b*+1, *N∗*10+*b*+2,…, *N∗*10+*b*+*T*(*b*), *b* = 1, 2, 3,…, *B*. *T*^(*b*, *j*)^ diseases are related to the disease type (*N∗*10+*b*)*∗*10+*j* and numbered as ((*N∗*10+*b*)*∗*10+*j*)*∗*10+1, ((*N∗*10+*b*)*∗*10+*j*)*∗*10+2,…, ((*N∗*10+*b*)*∗*10+*j*)*∗*10+*T*^(*b*, *j*)^, *b*=1,2,3,…, *B*, *j*=1,2,3,…, *T*(*b*).

Establish a data relationship list, in which the data structure is (Symptom 1, Symptom 2, Symptom 3,…, Symptom *N*, Disease). Each entry contains *N* symptoms. If symptom *n* does exist in the item of a disease, the value below “Symptom *n* ” is 1, or else, the value is 0.

For example, suppose that there are only *N*=11 symptoms in the current medical study records, the symptoms are male, fever, ulcer, pain, aching and limp, nasal congestion, diarrhea, bleeding, tumor, drowsiness, and face yellowing, and the label values of these symptoms are 1, 2, 3, 4, 5, 6, 7, 8, 9, 10, and 11. There are only *B*=10 major disease categories in the studied medical records, tumor disease, infectious disease, blood disease, cardiovascular disease, digestive disease, endocrine system disease, respiratory disease, urinary system disease, ophthalmic disease, and otolaryngology disease, and labelled numbers of these disease types are 101(*N∗*10+1), 102(*N∗*10+2), 103(*N∗*10+3), 104(*N∗*10+4), 105(*N∗*10+5), 106(*N∗*10+6), 107(*N∗*10+7), 108(*N∗*10+8), 109(*N∗*10+9), 110(*N∗*10+10), respectively. Furthermore, suppose that there are *T*(1)=3 subtype diseases, benign tumor 1011((*N∗*10+1)*∗*10+1), borderline tumor 1012((*N∗*10+1)*∗*10+2), and malignant tumor 1013((*N∗*10+1)*∗*10+3) in tumor diseases. And *T*^(1,1)^=5 diseases, which are squamous cell carcinoma 10111(((*N∗*10+1)*∗*10+1)*∗*10+1), adenocarcinoma 10112(((*N∗*10+1)*∗*10+1)*∗*10+2), basal cell carcinoma 10113(((*N∗*10+1)*∗*10+1)*∗*10+3), transitional cell carcinoma 10114(((*N∗*10+1)*∗*10+1)*∗*10+4) and sarcoma 10115(((*N∗*10+1)*∗*10+1)*∗*10+5), are in the benign tumor disease. If there is a medical record about the squamous cell carcinoma disease, and the symptoms are fever, ulcers, pain, and tumor, there are three data items that are related to this case and shown in Table 1.

The article "Intelligent Disease Prediagnosis Only Based on Symptoms" was published in 2021. Journal: J Healthc Eng.

A BP neural network that is shown in Figure 1 is used for the disease type and specific disease identification. There are *N* input layer nodes, Γ output layer nodes, and $Y=10+\sqrt{N+\Gamma }$ hidden layer nodes. *K* training symptom samples *o*(*k*)=(*x*_*k*_, *d*_*k*_), *k*=1,2,3,…, *K* are known. One medical record is related to a sample. When symptom *x*_*n*_^(*k*)^ appears in the record *x*^(*k*)^, *x*_*n*_^(*k*)^=1, or else *x*_*n*_^(*k*)^=0. When a medical record is about the disease type *d*_*ς*_^(*k*)^, *d*_*ς*_^(*k*)^=1, and the rest items are zero, that is, *d*_*q*≠*ς*_^(*k*)^=0. The (*N*+1) th input layer unit with an input value “−1” and the (*Y*+1)th hidden layer unit also with an input value “−1” are used to generate threshold values, and connection weights *ω*_(*N*+1)*p*_ and ${\overset{–}{\omega }}_{\left(Y+1\right)q}$ are used as thresholds *b*_*p*_ and *θ*_*q*_, respectively.

Specific training procedures are implemented according to formulas (1)–(13) in Section 3.2. Based on the data form in Table 1, the value of *x*_*n*_^(*k*)^ is 0 or 1, *n*=1,2,…, *N*. If *d*_*j*_^(*k*)^ is in {(*N∗*10+1), (*N∗*10+2),…, (*N∗*10+*B*)}, it is the training procedure to identify main disease categories. An identification neural network NT is obtained. If *d*_*j*_^(*k*)^ is in {(*N∗*10+*b*)*∗*10+1, (*N∗*10+*b*)*∗*10+2,…, (*N∗*10+*b*)*∗*10+*T*(*b*)}, it is the training procedure to identify subclass disease types under the main disease category *N∗*10+*b*. Identification neural networks NT − *b*, *b*=1,2,3,…, *B* are obtained. If *d*_*j*_^(*k*)^ is in {((*N∗*10+*b*)*∗*10+*j*)*∗*10+1, ((*N∗*10+*b*)*∗*10+*j*)*∗*10+2,…, ((*N∗*10+*b*)*∗*10+*j*)*∗*10+*T*^(*b*, *j*)^}, it is the training procedure to identify specific diseases under the subclass disease type (*N∗*10+*b*)*∗*10+*j*. Identification neural networks NT − (*b*, *j*), *b*=1,2,3,…, *B*, *j*=1,2,3,…, *T*(*b*) are obtained.

While the SVM method mentioned in Section 3.3 is used, classification parameters with respect to major disease types

(18) $$\begin{array}{c} {\left(\omega ,c\right)}^{1},{\left(\omega ,c\right)}^{2},\ldots ,{\left(\omega ,c\right)}^{B}, \end{array}$$

classification parameters with respect to subcategory disease types

(19) $$\begin{array}{c} {\left(\omega ,c\right)}^{\left(1,1\right)},{\left(\omega ,c\right)}^{\left(1,2\right)},\ldots ,{\left(\omega ,c\right)}^{\left(1,T\left(1\right)\right)},{\left(\omega ,c\right)}^{\left(2,1\right)},{\left(\omega ,c\right)}^{\left(2,2\right)},\ldots ,{\left(\omega ,c\right)}^{\left(2,T\left(2\right)\right)},\\ \cdots \\ {\left(\omega ,c\right)}^{\left(B,1\right)},{\left(\omega ,c\right)}^{\left(B,2\right)},\ldots ,{\left(\omega ,c\right)}^{\left(B,T\left(B\right)\right)}. \end{array}$$

and classification parameters with respect to specific diseases

(20) $$\begin{array}{c} {\left(\omega ,c\right)}^{\left(1,1,1\right)},{\left(\omega ,c\right)}^{\left(1,1,2\right)},\ldots ,{\left(\omega ,c\right)}^{\left(1,1,T^{\left(1,1\right)}\right)},{\left(\omega ,c\right)}^{\left(1,2,1\right)},{\left(\omega ,c\right)}^{\left(1,2,2\right)},\ldots ,{\left(\omega ,c\right)}^{\left(1,2,T^{\left(1,2\right)}\right)},\\ \cdots \\ {\left(\omega ,c\right)}^{\left(B,T\left(B\right),1\right)},{\left(\omega ,c\right)}^{\left(B,T\left(B\right),2\right)},\ldots ,{\left(\omega ,c\right)}^{\left(B,T\left(B\right),T^{\left(B,T\left(B\right)\right)}\right)}, \end{array}$$

can be obtained.

The article "Intelligent Disease Prediagnosis Only Based on Symptoms" was published in 2021. Journal: J Healthc Eng.

## 5. Diagnosis Implementations

### 5.1. Identification of Main Disease Categories

The symptoms, which are provided by a patient, are **κ**=(*κ*_1_, *κ*_2_,…, *κ*_*N*_).

1. Identification based on the neutral network: put **κ** into the neutral network NT to estimate which main disease category the symptoms refer to
2. Identification based on SVM: identify whether the disease category is based on vectors (**ω**, *c*)^*b*^, *b*=1,2,3,…, *B* by SVM

### 5.2. Identification of Subclass Disease Types

If the main disease category is *b*=*ς* and the symptoms provided by a patient are **κ**=(*κ*_1_, *κ*_2_,…, *κ*_*N*_), based on the neutral network NT − *ς* and SVM identification parameters (**ω**, *c*)^(*ς*, *τ*)^, *τ*=1,2,3,…, *T*(*ς*) to identify subclass disease types.

1. Subclass disease type identification based on the neutral network
2. Put **κ**=(*κ*_1_, *κ*_2_,…, *κ*_*N*_) into the neutral network NT − *ς* to estimate which subclass disease type the symptoms refer to.
3. Subclass disease type identification based on SVM
4. Step 1: Initial value is *τ*=1.
5. Step 2: Identify whether the disease type is *τ* based on vector (**ω**, *c*)^(*ς*, *τ*)^ in the SVM classification method. If the disease type is *τ*, go to Step 3, or else, make *τ*=*τ*+1. Verify that whether *τ* > *T*(*ς*), and if it is, quit out the whole procedure, or else loop through Step 2.
6. Step 3: The subclass disease type *τ* is the output result.

The article "Intelligent Disease Prediagnosis Only Based on Symptoms" was published in 2021. Journal: J Healthc Eng.

### 5.3. Identification of Specific Diseases

Suppose that the main disease category is *b*=*ς* and the subclass type is *j*=*τ*. Based on the neutral network NT − (*ς*, *τ*) and SVM identification parameters (**ω**, *c*)^(*ς*, *τ*, *υ*)^, *υ*=1,2,3,…, *T*^(*ς*, *τ*)^ to identify specific diseases.

1. Disease identification based on the neural network
2. Put **κ**=(*κ*_1_, *κ*_2_,…, *κ*_*N*_) into the neutral network NT − (*ς*, *τ*) to estimate what disease it is.
3. Disease identification based on SVM
4. Step 1: Initial value is *υ*=1.
5. Step 2: Identify whether the disease is *υ* based on vector (**ω**, *c*)^(*ς*, *τ*, *v*)^ in the SVM classification method. If the disease is *υ*, go to Step 3, or else make *υ*=*υ*+1. Verify that whether *υ* > *T*^(*ς*, *τ*)^, and if it is, quit out the whole procedure, or else loop through Step 2.
6. Step 3: Disease *υ* is the output result.

## 6. Method Tests

In this part, the diagnosis methods are tested. The tests in this paper are implemented in digestive diseases, respiratory diseases, and urinary diseases and used as examples.

### 6.1. Leave-One-Out Cross Validation

The neural network disease identification method and the support vector machine (SVM) disease identification method are compared.

**Example 1 .**

If a test sample is given, distinguish it as a digestive disease, a respiratory disease, or a urinary disease. Test results are shown in Table 2.

In Table 2, the accuracy of the main disease category identification is 94.4%.

Disease triage is to estimate which subclass disease type consulting symptoms provided by the user refer to. Disease triage is tested in the following examples.

**Example 2 .**

Tests are implemented in cases. Case 1: if a test sample has been diagnosed as a respiratory disease, distinguish it as a pulmonary disease, a respiratory tract infection, a chest disease, or a mediastinal disease. Case 2: if a test sample has been diagnosed as a digestive disease, distinguish it as an intestinal disease, a hepatic and gall disease, an epityphlon and pancreas disease, or a stomach disease. Case 3: If a test sample has been diagnosed as a urinary system disease, distinguish it as a bladder disease, a kidney disease, or an ureteral disease. The results are shown in Table 3.

In Table 3, the accuracy in disease subtype identification is higher than 80%, but lower than the accuracy in the main disease category identification.

Specific disease identification tests are carried on in Example 3 and Example 4. In Example 3, binary classification tests are executed. Samples about a disease are one class, samples not related to this disease are “the other” one. Example 4 is a multiclassification test, and samples related to different diseases are different categories.

The article "Intelligent Disease Prediagnosis Only Based on Symptoms" was published in 2021. Journal: J Healthc Eng.

**Example 3 .**

Tests are implemented in such cases. Case 1: Gastritis identification in stomach diseases; Case 2: Duodenal ulcer identification in stomach diseases. Case 3: Common cold identification in respiratory tract infections. Case 4: Pharyngitis disease identification in respiratory tract diseases; Case 5: Asthma identification in respiratory tract diseases. Case 6: Pneumonia identification in pulmonary diseases. Case 7: Pulmonary tuberculosis identification in pulmonary diseases. Case 8: Enteritis identification in intestinal diseases. Case 9: Intestinal obstruction identification in intestinal diseases. Case 10: Hepatitis identification in hepatic and gall diseases. Case 11: Gallstone identification in hepatic and gall diseases. Test results are shown in Table 4.

**Example 4 .**

Tests are implemented in such cases: Case 1: Gastritis, upper gastrointestinal bleeding, duodenal ulcer, and gastric ulcer identifications in stomach diseases; Case 2: Intestinal obstruction, intussusception, ulcerative colitis, common enteritis, and lower gastrointestinal bleeding identifications in intestinal diseases; Case 3: Viral hepatitis, cholangitis, gallstones, cholecystitis, liver abscess, and cirrhosis identifications in hepatic and gall diseases; Case 4: Pneumonia, emphysema, lung abscess, pulmonary thrombosis, and tuberculosis identifications in pulmonary diseases; Case 5: Upper respiratory tract infection and lower respiratory tract infection identifications in respiratory tract infections; Case 6: Renal failure, glomerulonephritis, pyelonephritis, kidney stones, and nephrotic syndrome identifications in kidney diseases. Test results are shown in Table 5.

Comparing the results in Tables 4 and 5, if the specific disease diagnosis is put into binary classifications, the accuracy is higher than 80%, and when it is put into multiclassification modules, the results are unsatisfactory. Without the support of detailed pathology data, specialized diseases actually cannot be accurately diagnosed by methods only based on symptoms. However, considering the result supports in Table 4, identifications of common diseases such as gastritis, common cold, pharyngitis, and common enteritis, which always do not need the support of detailed pathology data, can be provided to the user in an automatic disease diagnosis system.

### 6.2. Diagnosis with Weight Samples

In clinic, some diseases have high relational discrepancy symptoms. In a common disease diagnosis experiment, which we have carried out, sample weights are assigned to some samples artificially according to clinical experience, and these weights are added into loss functions in machine learning procedures [17]. In the test, binary classification results using samples with weights and without weights are similar, and the precision difference is less than 4%. Thus, high relational discrepancy degree samples are suggested to be put into test sample sets in validation procedures of machine learning methods.

The article "Intelligent Disease Prediagnosis Only Based on Symptoms" was published in 2021. Journal: J Healthc Eng.

### 6.3. Multitype Diseases Diagnosis

A person may have more than 1 disease, and these diseases refer to different types, and results also can be obtained when **κ**=(*κ*_1_, *κ*_2_,…, *κ*_*N*_) is put into classification modules identifying 1, 2, 3,…, *N* concurrence diseases successively.

**Example 5 .**

Suppose that a patient has two or three diseases, and these diseases belong to different disease subtypes. Case 1: If the diseases belong to digestive diseases, identify it as a concurrence case of intestinal disease, and hepatic and gall disease, a concurrence case of intestinal disease and stomach disease, or a concurrence case of stomach disease, and hepatic and gall disease. Case 2: If the diseases belong to respiratory diseases, identify it as a concurrence case of pulmonary disease and chest disease, a concurrence case of chest disease and respiratory tract infection, or a concurrence case of pulmonary disease and respiratory tract infection. Case 3: If the diseases belong to respiratory diseases, identify it as a concurrence case of pulmonary disease, upper respiratory tract disease, and trachea and bronchi disease, a concurrence case of pulmonary disease, upper respiratory tract disease, and pleura and chest disease, or a concurrence case of pulmonary disease, trachea and bronchi disease, and pleura and chest disease. Case 4: If the diseases belong to digestive diseases, identify it as a concurrence case of intestinal disease, hepatic and gall disease, and epityphlon and pancreas disease, a concurrence case of stomach disease, intestinal disease, and hepatic and gall disease, or a concurrence case of epityphlon and pancreas disease, stomach disease, and intestinal disease. The above cases are about disease subtype identifications, and the results are shown in Table 6.

From the results in Table 6, it can be seen that, in the identification of concurrence of multiple disease types, the accuracy of machine learning methods is dropping. When there is a concurrence of more than three disease types, the identification accuracy would be much lower.

### 6.4. Discussion on Test Results

1. For lacking pathologic support, the accuracy of the GP diagnosis methods based on symptoms for specific diseases is limited. In our tests, it is shown that this kind of methods can be used in the diagnosis of common diseases, such as cold, enteritis, and rhinitis, and for specialized diseases such as asthma, liver cancer, and psoriasis, these methods can be used to predict disease types and provide disease triage. Diagnosis methods, which identify disease types in this paper, can also be used in hospital guides.
2. In consideration of sample characteristics, the neutral network and SVM machine learning methods are appropriate choices for the automatic prediagnosis problem in this paper. In our experiments, the accuracy of the neural network is close to that of SVM. Sometimes, the neutral network performs a litter better, and sometimes, it is the SVM. A corollary is that the accuracy of this kind of diagnosis methods is limited by the problem itself, and even another practicable machine learning method is adopted, and the performance is also similar with the neutral network and SVM method.
3. From the experiment results, it can be seen that automatic prediagnosis methods only based on symptom data are suitable for single disease type identification, and it is also not difficult to infer that these methods are also only suitable for a specific common disease identification. If a symptom record is related to multiple disease types or multitype diseases, the availability is low.
4. In our experiments, the feasibilities of diagnosis only based on symptoms using machine learning methods are tested. Even tests are carried out in digestive diseases, respiratory diseases, and urinary diseases, and without loss of generality, it can be deduced that this kind of diagnosis methods can be used in other disease categories. Test results would also be observed further in more kinds of disease types except for the cases in this paper.

The article "Intelligent Disease Prediagnosis Only Based on Symptoms" was published in 2021. Journal: J Healthc Eng.

## 7. Conclusions

In this paper, neural network and SVM machine learning methods are given to solve the automatic disease diagnosis problem only based on symptoms. In our methods, each symptom is a feature. The methods work in three layers, which are main disease category identification, subclass disease type identification, and specific disease identification. The methods are suitable for the diagnosis of common diseases and disease triage for specialized diseases. The availability in practice is proved and analyzed in the experiments of this paper. In addition, future research is also required to investigate automatic symptom extraction and discuss the maximum number size of symptoms.

## Figures and Tables

**Figure 1:** BP neural network in this paper.

**Table 1:** An example of disease records.

Sequence number	Gender	Fever	Ulcer	Pain	Aching and limp	Nasal congestion	Diarrhea	Bleeding	Tumor	Drowsiness	Face yellowing	Disease
1	1	1	1	1	0	0	0	0	1	0	0	101
2	1	1	1	1	0	0	0	0	1	0	0	1013
3	1	1	1	1	0	0	0	0	1	0	0	10131

**Table 2:** Diagnosis of main disease categories.

Number of test samples	Wrong identified samples	Methods
169	9	SVM
169	9	Neural network

**Table 3:** Disease triage.

Cases	Number of test samples	Wrong identified samples	Methods
Case 1	76	15	SVM
	76	15	Neural network

Case 2	60	12	SVM
	60	11	Neural network

Case 3	32	4	SVM
	32	4	Neural network

**Table 4:** Diagnosis of specific diseases in binary classifications.

Cases	Accuracy (%)	Methods
Case 1	80.48	SVM
	82.93	Neural network

Case 2	85.36	SVM
	85.36	Neural network

Case 3	91.43	SVM
	88.57	Neural network

Case 4	97.14	SVM
	97.14	Neural network

Case 5	88.00	SVM
	88.00	Neural network

Case 6	80.00	SVM
	84.00	Neural network

Case 7	80.00	SVM
	80.00	Neural network

Case 8	86.00	SVM
	86.00	Neural network

Case 9	88.00	SVM
	90.00	Neural network

Case 10	95.00	SVM
	93.33	Neural network

Case 11	83.33	SVM
	83.33	Neural network

**Table 5:** Diagnosis of specific diseases in multiple classifications.

Cases	Accuracy (%)	Methods
Case 1	41.46	SVM
	34.15	Neural network

Case 2	78.00	SVM
	70.00	Neural network

Case 3	66.67	SVM
	63.33	Neural network

Case 4	60.00	SVM
	56.00	Neural network

Case 5	76.00	SVM
	70.00	Neural network

Case 6	70.00	SVM
	60.00	Neural network

**Table 6:** Diagnosis of multiple diseases.

Cases	Number of test samples	Wrong identified samples	Methods
Case 1	150	54	SVM
	150	52	Neural network

Case 2	150	36	SVM
	150	36	Neural network

Case 3	180	135	SVM
	180	133	Neural network

Case 4	200	134	SVM
	200	136	Neural network

## Data Availability

The data used to support the findings of this study are included within the supplementary information file.

## Supplementary Materials

Supplementary Materials Data file “prototype data.pdf.”
